The article "Metformin in Combination with Progesterone Improves the Pregnancy Rate for Patients with Early Endometrial Cancer" was published in 2022. Journal: Contrast Media Mol Imaging.

# Metformin in Combination with Progesterone Improves the Pregnancy Rate for Patients with Early Endometrial Cancer

**DOI:** 10.1155/2022/1961016

**Published:** 2022-07-06

**Authors:** Feng Yuan, Ying Hu, Xi Han, Qiumin Li

**Affiliations:** Department of Obstetrics, Shaanxi Provincial People's Hospital, Xi'an, China

## Abstract

*Objective*. To study the therapeutic effects of metformin in combination with medroxyprogesterone in the early endometrial cancer patients with fertility requirements. A total of 120 patients with early endometrial cancer admitted to and treated in our hospital were enrolled and evenly assigned into two groups according to different therapeutic regimens, namely, metformin group (metformin combined with medroxyprogesterone acetate) and control group (medroxyprogesterone acetate alone). The objective response rate (ORR) and disease control rate (DCR) were 71.7% (43/60) and 90.0% (54/60) in the metformin group and 53.3% (32/60) and 78.3% (47/60) in the control group, respectively. Adverse reactions such as gastrointestinal reaction, headache, and insomnia were mainly observed in patients. The body mass index (BMI) declined from (34.43 ± 4.34) kg/m^2^ to (24.77 ± 2.39) kg/m^2^ in the metformin group and from (33.37 ± 4.49) kg/m^2^ to (31.28 ± 3.55) kg/m^2^ in the control group after treatment. After treatment, serum levels of vascular endothelial growth factor (VEGF), angiotensin-2 (Ang-2), carbohydrate antigen 125 (CA125), and CA19-9 in the metformin group were significantly lower than those in the control group (*P* = 0.005, *P* < 0.001, *P* = 0.002, and *P* < 0.001). During follow-up, the pregnancy rate was 81.7% (49/60) in the metformin group and 61.7% (37/60) in the control group, and the former was prominently higher than the latter (*P* = 0.025). Metformin in combination with progesterone is effective in treating early endometrial cancer patients with fertility requirements, which significantly reduced the BMI of patients and increased the pregnancy rate after treatment.

## 1. Introduction

Endometrial cancer, one of the most common cancers of female reproductive system, accounts for about 7% of malignant tumors in females. Its incidence rate rises obviously in females aged below 40 years old in recent years, which is about 2–14% and increasing year by year [1]. Among such patients, 70% are nulliparous, so preserving the fertility function is of importance. Surgical resection is effective in the treatment of endometrial cancer, whose standard surgical approach is total hysterectomy + bilateral salpingo-oophorectomy, as well as lymph node dissection according to the clinical stage of patients. As a result, patients will permanently lose fertility [2].

The article "Metformin in Combination with Progesterone Improves the Pregnancy Rate for Patients with Early Endometrial Cancer" was published in 2022. Journal: Contrast Media Mol Imaging.

Progesterone therapy is a therapeutic method most commonly used in clinic to preserve the fertility of patients. However, adverse reactions including progesterone resistance, thrombosis, and weight gain are observed with increasing application in clinical practice, affecting the treatment efficacy and compliance of patients [3, 4]. Metformin, a first-line drug for the treatment of diabetes, has been proven in many studies to be able to reduce the incidence rate, progression, and mortality rate of different human cancers, including EC [5]. Besides, previous evidence has demonstrated that metformin can increase progesterone sensitivity and improve progesterone resistance [6–9]. In the present research, the therapeutic effect of metformin in combination with progesterone in treating early endometrial cancer with fertility requirements was investigated, hoping to offer a basis for clinical research.

## 2. Materials and Methods

### 2.1. General Data

The clinical data of 120 patients with early endometrial cancer admitted to and treated in our hospital were collected (the trial registration number: ChiCTR1800020281) (Table 1). The inclusion criteria were set as follows:

1. Endometrioid well-differentiated adenocarcinoma diagnosed by histopathological examination after operation.
2. Patients with involved myometrium <1/2 and no extra-uterine lesions and lymph node metastasis by MRI.
3. Those who were aged <40 years old, nulliparous, and still had the willingness to bear children.
4. Those with estrogen-dependent and progesterone receptor (PR)-positive endometrial cancer.

The exclusion criteria were as follows:

1. Those who received other anti-tumor therapy were excluded.
2. Patients with severe heart, lung, liver, and kidney dysfunction, coagulation dysfunction, immune system disorders, or infectious diseases.
3. Patients with other malignant tumors.
4. Patients with abnormal neurological function.

The enrolled patients were divided into two groups according to different therapeutic regimens, namely, metformin group (metformin combined with medroxyprogesterone acetate, *n* = 60) and control group (medroxyprogesterone acetate alone, *n* = 60). Written signed informed consent was obtained from each patient before the study. This study was approved by the ethical committee of our hospital.

### 2.2. Therapeutic Methods

Patients in the control group took medroxyprogesterone acetate dispersible tablets (manufactured by Nanjing Cuccess Pharmaceutical Co., Ltd., Nanjing, China) orally at 0.4–0.8 g/d. In the metformin group, metformin (manufactured by Changzhou Pharmaceutical Factory Co., Ltd., Changzhou, China) was administrated orally (0.5 g/time, 3 times/d) in addition to the treatment in the control group. During continuous treatment, the clinical symptoms of patients in the two groups were closely observed. Administration was stopped when no residual disease was found. Patients could get pregnant only after 3 months of drug withdrawal.

The article "Metformin in Combination with Progesterone Improves the Pregnancy Rate for Patients with Early Endometrial Cancer" was published in 2022. Journal: Contrast Media Mol Imaging.

### 2.3. Observation Indexes

The following indicators were calculated: complete remission (CR): lesions disappeared, with atrophy of endometrial glands and decidual response in the stroma, partial remission (PR): there were residues of hyperplastic endometrium, without atypical cell residues, stable disease (SD): histopathological examination results were consistent with those before treatment, and progressive disease (PD): myometrial infiltration was deepened or metastasis appeared. Objective response rate (ORR) = (CR + PR)/total number of cases  ×  100%; disease control rate (DCR) = (CR + PR + SD)/total number of cases  ×  100%.

The levels of tumor markers, including vascular endothelial growth factor (VEGF), angiotensin-2 (Ang-2), carbohydrate antigen (CA) 125, and CA19-9, were evaluated. Besides, the body mass index (BMI) of patients was also analyzed, and the incidence rate of adverse reactions such as gastrointestinal reactions, insomnia, and headache was compared between the two groups of patients.

Besides, the successful pregnancy rate, pregnancy status, and pregnancy outcome of patients in the two groups were followed up and recorded.

### 2.4. Statistical Analysis

SPSS 19.0 software (IBM, Armonk, NY, USA) was used for statistical analyses. All quantitative data were expressed as mean ± standard deviation. Student's *t*-test was employed for comparing the variables before and after treatment. Percentage (%) was used to express the enumeration data, and the chi-square test was used for data analysis. A significant difference was set at *P* < 0.05.

## 3. Results

### 3.1. Comparison of Clinical Efficacy in Patients

The efficacy was assessed after treatment of all patients. The ORR and DCR were 71.7% (43/60) and 90.0% (54/60) in the metformin group and 53.3% (32/60) and 78.3% (47/60) in the control group, respectively. The ORR was remarkably higher in the metformin group than the control group (*P* = 0.038), whereas the DCR had no statistically significant difference (*P* = 0.132) (Table 2).

### 3.2. Evaluation of Adverse Reactions

Adverse reactions such as gastrointestinal reactions, headaches, and insomnia were mainly observed in patients. There were 8 (13.3%) and 5 (8.3%) cases of gastrointestinal reactions, 6 (10.0%) and 6 (10.0%) cases of headache, 5 (8.3%) and 5 (8.3%) cases of insomnia in the metformin group and control group, respectively.

The article "Metformin in Combination with Progesterone Improves the Pregnancy Rate for Patients with Early Endometrial Cancer" was published in 2022. Journal: Contrast Media Mol Imaging.

### 3.3. Comparisons of BMI and Serum VEGF, Ang-2, CA125, and CA19-9 Levels

The BMI declined from (34.43 ± 4.34) kg/m^2^ to (24.77 ± 2.39) kg/m^2^ in the metformin group and from (33.37 ± 4.49) kg/m^2^ to (31.28 ± 3.55) kg/m^2^ in the control group after treatment. The serum VEGF, Ang-2, CA125, and CA19-9 levels displayed no statistically significant differences (*P* = 0.299, *P* = 0.580, *P* = 0.376, and *P* = 0.377). After treatment, such levels declined in both groups (VEGF: (482.31 ± 23.67) ng/L and (477.97 ± 21.89) ng/L to (287.63 ± 25.85) ng/L and (302.51 ± 30.43) ng/L, Ang-2: (1.47 ± 0.40) *μ*g/L and (1.51 ± 0.39) *μ*g/L to (0.39 ± 0.09) *μ*g/L and (0.45 ± 0.11) *μ*g/L, CA125: (53.03 ± 6.11) U/mL and (52.08 ± 5.58) U/mL to (28.78 ± 3.03) U/mL and (30.29 ± 2.21) U/mL, and CA19-9: (22.82 ± 1.96) kU/L and (22.49 ± 2.11) kU/L to (10.47 ± 1.08) kU/L and (12.63 ± 3.05) kU/L) (Figure 1).

### 3.4. Pregnancy Outcomes

Results showed that the pregnancy rate was 81.7% (49/60) in the metformin group and 61.7% (37/60) in the control group. Naturally pregnant patients accounted for 67.3% (33/60) and 62.2% (23/60) of the total pregnant patients, and patients who got pregnant by assisted reproductive technology accounted for 32.7% (16/60) and 37.8% (14/60) of the total pregnant patients in metformin and control groups. Abortion, premature delivery, and term delivery were found in 8.2% and 10.8%, 16.3% and 18.9%, and 75.5% and 70.3% of pregnant patients in metformin and control groups, respectively (Table 3).

## 4. Discussion

Generally, the attack of early endometrial cancer in young patients has associations with factors such as obesity, insulin resistance, ovulation disorders, and infertility [10]. Studies have manifested that obesity and insulin resistance are related factors for the high recurrence rate and long duration of conservative treatment of endometrial cancer [11, 12]. For this reason, alleviating obesity, insulin resistance, and other metabolic syndromes in patients will be a new strategy for the conservative treatment of endometrial cancer. In recent years, metformin, an insulin sensitizer, has been applied by researchers in the conservative treatment of endometrial cancer. The study findings have shown that metformin can improve the effect of conservative treatment to some extent [13, 14].

A phase II clinical trial conducted by Mitsuhashi et al. in 2015, in which 36 patients with atypical endometrial hyperplasia/endometrial cancer (stage I, G1) were treated with MPA in combination with metformin for 24–36 weeks, reported that CR is found in 81% (29/36) of patients within 36 weeks, with a median follow-up of 38 months, and recurrence is observed in only 3 patients [15]. It was discovered in another study where the long-term efficacy of MPA combined with metformin conservative treatment was evaluated that the 12 and 18-month CR rates are 90% and 97%, respectively, with a median follow-up of 57 months, the recurrence rate is only 13%, and more benefits are obtained by obese patients from metformin-based combined therapy. It is probably because that metformin suppresses the secretion of adipokines, the driving factors for the increased obesity-induced risk of endometrial cancer, from adipocytes [16].

The article "Metformin in Combination with Progesterone Improves the Pregnancy Rate for Patients with Early Endometrial Cancer" was published in 2022. Journal: Contrast Media Mol Imaging.

To find out whether metformin in combination with progesterone has a better therapeutic effect than progesterone alone, a study was conducted on 120 patients with early endometrial cancer. The results uncovered that the 16-week CR rate is higher in metformin + MA group than that in MA group. It was found through sub-group stratified analysis that patients with atypical dysplasia benefit more from metformin: the 16-week CR rate in metformin + MA group is almost twice that in MA group. Additionally, obese and insulin-sensitive patients also benefit from it [17]. However, a recent study reported that the recurrence rate shows no statistically significant difference between metformin combined with progesterone and progesterone alone (17% *vs.* 25%, *P* = 0.484). In the above-mentioned study, the BMI of patients is higher in metformin treatment group than that in control group (*p* = 0.042), and the dose of metformin is 500–1,000 mg. The insufficient dose of metformin and the heterogeneity of BMI between treatment groups may have some influence on the results of the study, so further research should be carried out for verification [18]. A meta-analysis by Chae-Kim et al. demonstrated that the combination therapy of progesterone and metformin is associated with lower relapse rates and similar remission, clinical pregnancy, and live birth rates for reproductive-aged women with atypical endometrial hyperplasia or early endometrial cancer [19]. Existing studies have manifested that metformin improves the remission rate and reduces the recurrence rate of conservatively treated patients to some extent. The results of this study revealed that the ORR was significantly higher in the metformin group than that in the control group, suggesting that metformin in combination with progesterone gets better therapeutic results than progesterone alone in patients with endometrial cancer.

Usually, conservative treatment with progesterone is adopted to alleviate tumor progression, conducive to pregnancy. The meta-analysis by Koska et al. showed that the pregnancy rate is 32% (111/351) after conservative treatment of endometrial cancer, implying that the traditional progesterone therapy leads to a poor pregnancy outcome. Hence, discovering new strategies to change this situation is urgent [20]. Considering that patients with endometrial cancer often suffer from infertility factors like obesity, polycystic ovary syndrome, and ovulation disorders, relieving the abnormal metabolism of their body may be a new direction for treatment. Research shows that metformin can attenuate ovulation disorders and promote pregnancy by improving the insulin resistance, glucose intolerance, and other metabolic status of patients with polycystic ovary syndrome [21]. In recent years, the application of metformin in the conservative treatment of endometrial cancer has been widely studied, and the results revealed that metformin is able to improve the pregnancy outcomes of patients. A study by Mitsuhashi et al. reported that CR is achieved through treatment with metformin combined with MPA, 50% (8/16) of early endometrial cancer patients who tried to get pregnant (16/29) are successfully pregnant, and the live birth rate is 37.5% [10]. It was found in another retrospective study that the overall pregnancy rate is 61% (19/31) after metformin combined with progesterone conservative treatment, and the live birth rate is 45% (14/31) [16]. According to a recent prospective randomized controlled trial by Yang et al., the pregnancy rate is 51.8% in metformin + MA group (*n* = 37) and 48.4% in MA group (*n* = 31) [17]. The above findings indicate that the application of metformin improves the pregnancy rate of patients to a certain extent. It was found in this study that during follow-up, the pregnancy rate was significantly higher in the metformin group than that in the control group (81.7% *vs.* 61.7%, *P* = 0.025), and the metformin group also had a higher proportion of natural pregnancy than the control group, but the difference was of no statistical significance. It implies that metformin improves the pregnancy outcome of patients to some extent. The main novelty of the present study was that the patients enrolled in this research were evaluated comprehensively, including the clinical efficacy, adverse reactions, tumor marker levels, pregnancy rate, and abortion results. However, limitations also existed in this study. The limited sample size, short follow-up time, and incomprehensive follow-up content might lead to the biased conclusions. Prospective clinical research data with rigorous design, high reliability, and large sample size are needed to support the conclusions drawn in this study in the future.

The article "Metformin in Combination with Progesterone Improves the Pregnancy Rate for Patients with Early Endometrial Cancer" was published in 2022. Journal: Contrast Media Mol Imaging.

## 5. Conclusion

Metformin in combination with progesterone has exact effects in treating early endometrial cancer patients with fertility requirements, which is capable of significantly decreasing the BMI of patients and elevating the pregnancy rate after treatment.

## Figures and Tables

**Figure 1:** Evaluation of the serum markers of the patients in the 2 groups: VEGF (a), Ang-2 (b), CA125 (c), and CA19-9 (d) (^*∗*^*p* < 0.05).

**Table 1:** Demographic characteristics of the patients in the 2 groups.

Indicators	Metformin group (*n* = 60)	Control group (*n* = 60)	*P* value
Age (years)	33.73 ± 7.47	35.12 ± 8.41	0.257
BMI (kg/m^2^)	34.43 ± 4.24	33.37 ± 4.49	0.368
Irregular menstruation (*n*, %)	38 (63.3%)	43 (71.7%)	0.563
Course of disease (months)	10.3 ± 3.3	10.8 ± 3.6	0.437
PCOS (*n*, %)	21 (35.0%)	18 (30.0%)	0.578
Insulin resistance (*n*, %)	19 (31.7%)	17 (28.3%)	0.444

PCOS: polycystic ovary syndrome.

**Table 2:** Analysis of the therapeutic effects in patients of the two groups.

Indicators	Metformin group (*n* = 60)	Control group (*n* = 60)	*P* value
Complete response (CR)	16 (26.7%)	12 (20.0%)	
Partial response (PR)	27 (45.0%)	20 (33.3%)	
Stable disease (SD)	11 (18.3%)	15 (25.0%)	
Progressive disease (PD)	6 (10.0%)	13 (21.7%)	
ORR (CR + PR)	43 (71.7%)	32 (53.3%)	0.038
DCR (CR + PR + SD)	54 (90.0%)	47 (78.3%)	0.132

**Table 3:** Evaluation of the pregnancy outcomes of the patients.

Index	Metformin group (*n* = 60)	Control group (*n* = 60)	*P* value
Pregnancy rate (%)	49 (81.7%)	37 (61.7%)	0.025
Natural pregnancy	33 (67.3%)	23 (62.2%)	
ART pregnancy	16 (32.7%)	14 (37.8%)	
Pregnancy outcome			0.752
Abortion	4 (8.2%)	4 (10.8%)	
Premature delivery	8 (16.3%)	7 (18.9%)	
Term delivery	37 (75.5%)	26 (70.3%)	

ART: assisted reproductive technology.

## Data Availability

The datasets used and analyzed during the current study are available from the corresponding author on reasonable request.
